# The Efficacy of Psychological Care and Chinese Herbal Decoction in Postoperative Chemotherapy Patients with Endometrial Cancer

This article has been retracted.

**DOI:** 10.1155/2022/5700637

**Published:** 2022-02-18

**Authors:** Jinjie Liu, Juan Wang, Yang Guo, Hongmei Zhang

**Affiliations:** ^1^Medical Insurance Department, Zhangqiu District People's Hospital, Jinan 250200, Shandong Province, China; ^2^Department of Clinical Laboratory, Zhangqiu District People's Hospital, Jinan 250200, Shandong Province, China; ^3^Department of Gynaecology, Renzheng Hospital, Renzheng 265811, Shandong Province, China; ^4^PIVAS, Yantaishan Hospital, Yantai 264001, Shandong Province, China

## Abstract

**Background:**

In recent years, the incidence of endometrial cancer (EC) has been on the rise worldwide. The purpose of this study was to investigate the efficacy of psychological care and Chinese herbal decoction in EC patients with postoperative chemotherapy.

**Methods:**

80 EC patients with postoperative chemotherapy were randomly divided into the observation group and control group. The control group was given psychotherapy. The observation group was given psychological care plus Chinese herbal decoction treatment. HE4, CA125, traditional Chinese medicine (TCM) syndrome scores, toxic and side effects, and quality of life scores before and after treatment were observed.

**Results:**

After treatment, the total effective rate of the observation group was higher than that of the control group. After treatment, serum HE4 and CA125 levels in the observation group were lower than those in the control group. In addition, CD3+ and CD4+ levels in the observation group were higher than those in the control group. Meanwhile, the CD8+ level in the observation group was lower than that in the control group. Compared with the control group, the quality of life in the observation group was significantly improved, and the incidence of adverse reactions was reduced.

**Conclusion:**

Chinese herbal decoction combined with psychological care can improve the clinical symptoms, alleviate the toxic and side effects, and improve the life quality of EC patients with postoperative chemotherapy.

## 1. Introduction

Endometrial carcinoma (EC) is one of three common malignancies in the female reproductive system. The incidence of postmenopausal women in Western developed countries is higher, and the incidence of EC in developing countries is second only to cervical cancer [1, 2]. In recent years, decreased exercise and high-fat eating habits have led to an increase in obesity. Obesity can lead to polycystic ovary syndrome, infertility, and delayed menopausal age in women [3, 4]. These diseases lead to high incidence of EC, which seriously threaten women's health [5, 6]. At present, the clinical treatment of EC is mainly surgery combined with chemotherapy. Chemotherapy has certain curative effects, but it has serious side effects. Frailty and poor tolerance in EC patients lead to increased mortality [7, 8].

With the development of postoperative adjuvant chemotherapy, the therapeutic effect of EC has been improved to varying degrees. However, about 30% of patients remain at risk of recurrence and metastasis after treatment. As many as 60% of patients occur within 1 year, suggesting that the treatment of patients with recurrence and metastasis is also an urgent problem to be solved [9]. Adjuvant chemotherapy alone may not improve recurrence and metastasis in EC patients [10]. Therefore, while inhibiting disease progression, it is also necessary to improve the life quality of patients to improve their prognosis. The use of traditional Chinese medicine on the basis of conventional Western medicine and chemotherapy is beneficial to improve the life quality of patients with malignant tumors [11].

Traditional Chinese medicine believes that EC is a disorder of Yin and Yang caused by renal failure and exhaustion of Tiangui [12–14]. Traditional Chinese medicine treatment can reduce the side effects of radiotherapy and chemotherapy, improve the clinical symptoms of patients, and improve the life quality of patients [15–18]. On the basis of surgical treatment and chemotherapy, according to the patient's treatment effect and symptoms, Chinese medicine decoction can restore the patient's qi and blood and has a synergistic detoxification effect. Traditional Chinese medicine can eliminate tumor nodules or cancer cell residues, improve the patient's physical and mental symptoms, and improve the life quality and the body's disease resistance [19–23].

Recently, the role of comprehensive care in cancer treatment has gradually been paid more and more attention by clinicians [24–27]. There are many studies about the effect of psychological intervention on postoperative recovery in noncancer patients [28, 29]. Psychological nursing refers to the process of influencing the psychological activities, individual characteristics, or psychological problems of a certain object in a planned and step-by-step manner under the guidance of psychological theory. Therefore, effective postoperative psychological nursing intervention is of great significance for accelerating the recovery of patients and improving the patients' negative emotions and quality of life.

In order to seek effective methods to consolidate the effect of chemotherapy and adjuvant therapy to relieve discomfort, reduce functional damage, and improve the life quality, this study investigated the efficacy of psychological care and Chinese herbal decoction in EC patients with postoperative chemotherapy. Our study aimed to provide a symptom improvement method with proven efficacy, few side effects, and low cost for EC patients undergoing chemotherapy.

## 2. Materials and Methods

### 2.1. Patients

A total of 80 EC patients who met the inclusion criteria of this study from January 2018 to December 2019 were collected. The patients were divided into 2 groups by the random number table method (*n* = 40). There were no significant differences in age, weight, cancer stage, and pathological classification between the two groups (Table 1).

### 2.2. Inclusion and Exclusion Criteria

Inclusion criteria: EC confirmed by surgery and pathological biopsy, 42–69 years old, first surgery and chemotherapy, expected survival time >6 months, and patients and their guardians signed the informed consent. This study was approved by the Ethics Committee of Yantaishan Hospital.

Exclusion criteria: complicated with hematological diseases, other malignant tumors, and neurological diseases; allergic to the drugs used in this study; complicated infections, diabetes, hypertension, and immune system diseases; and activated partial thromboplastin time (APTT) exceeds the normal value 2 times. There is a tendency to bleed. Platelet count (BPC) is less than 60× 10^9^/L.

### 2.3. Treatment

The control group received conventional chemotherapy combined with nursing intervention. TP program: paclitaxel (135–175 mg/m^2^) was given intravenously for 3 h. After that, cisplatin (70 mg/m^2^) was injected. Dexamethasone was given as pretreatment before chemotherapy, and antiemetic, acid suppression, and fluid rehydration therapy were also given at the same time. All chemotherapy drugs were administered intravenously with an interval of 3 weeks for 4–6 courses.

The observation group was treated with traditional Chinese medicine on the basis of the control group. The prescription includes 30 g of *Astragalus*, 20 g of *Codonopsis*, 15 g of *Hedyotis diffusa*, 15 g of Shantou mushroom, 15 g of *Prunella vulgaris*, 12 g of *Angelica sinensis*, 15 g of trigonum, 12 g of turmeric, 10 g of corrugated seed, 0.05 g of cantharidin, 10 g of *Corydalis*, 12 g of *Citrus aurantium*, green peel 12 g, *Pinellia* 10 g, *Amomum* 6 g, raw malt 30 g, *Gallus Gallus domesticus* 20 g, *Asparagus* 15 g, *Ophiopogon* 15 g, Sichuan *Achyranthes* 10 g, and licorice 5 g. Each dose is decocted 3 times. The traditional Chinese medicine is provided to patients in 3 bags (200 mL, the quality standard refers to the standard requirements for oral liquid preparations of the 2020 edition of the Chinese Pharmacopoeia).

### 2.4. Serum Marker Detection

Serum tumor marker levels were detected 1 day before treatment and after 3 courses of treatment. 5 mL of fasting venous blood was taken from the patient and centrifuged at 3000 r/min for 10 minutes. The supernatant was aspirated into the EP tube using a pipette. Serum human epididymal protein 4 (HE4) and serum sugar chain antigen 125 (CA125) levels were detected by enzyme-linked immunosorbent assay (ELISA). ELISA was performed using an ARCHITECT i4000SR automatic immunoassay analyzer (Abbott, USA). Special matching kits were used in accordance with the kit instructions.

### 2.5. Immunoglobulin Detection

The changes of immunoglobulin *G* (IgG) and immunoglobulin A (IgA) in the two groups before and after treatment were observed. The levels of immunoglobulin IgG and IgA in peripheral blood of patients were detected by the flow cytometer using the fluorescent molecular labeling method.

### 2.6. Immune Function Test

CD3+, CD4+, and CD8+ were detected 1 day before and after treatment. The levels of peripheral blood T lymphocyte subsets were detected by the flow cytometer (CyFlow®Cube8, Partec, Germany) using the fluorescent molecular labeling method.

### 2.7. Evaluation Index

After treatment, the visual analogue scale (VAS) was used to evaluate postoperative pain in the two groups, with a total score of 0–10. The higher the score, the more severe the pain.

#### 2.7.1. Quality of Life

We used the patient's oral quality of life scores and recorded survival outcomes weekly after the patient's postoperative chemotherapy treatment [30].

#### 2.7.2. TCM Syndrome Score

The TCM syndrome scores of the two groups before and after treatment were observed. The lower the fatigue symptom score, the better. The higher the function score, the better.

#### 2.7.3. Adverse Reactions

Cancer-related symptoms or side effects of cancer treatment include pain, flushing, anorexia, fatigue, sleep disorders, negative emotions, lymphedema, neuropathy, oral ulcers, constipation or diarrhea, nausea, and vomiting. The Common Terminology Criteria for Adverse Events (CTCAE) scale was used [31].

### 2.8. Statistical Analysis

All experiments were performed in 3 replicates. Statistical analysis was performed using SPSS 22.0 software. Measurement data are expressed as mean ± standard deviation, and count data are expressed as *n* (%). Comparisons were made by the *χ*^2^ test. The difference was statistically significant when *P* < 0.05.

## 3. Results

### 3.1. Comparison of Tumor Marker Levels between the Two Groups

Before treatment, there was no significant difference in the levels of tumor markers HE4 and CA125 between the observation group and the control group (*P* > 0.05, Figure 1). After treatment, serum HE4 and CA125 levels in both groups were significantly lower than those before treatment (*P* < 0.05, Figure 1). The degree of decline in the observation group was higher than that in the control group, suggesting that chemotherapy-assisted psychological nursing intervention combined with Chinese medicine decoction treatment can improve the curative effect of EC patients.

### 3.2. Comparison of Blood Routine and Liver Function between Two Groups before and after Treatment

There was a statistically significant difference in red blood cell count (RBC, *P* < 0.05, Table 2) between the control group and the observation group. However, there were no significant changes in body weight between the two groups (Table 2). Liver damage caused by cancer treatment is common. It can be caused by certain chemotherapy drugs (carboplatin, etoposide, cisplatin, and paclitaxel), active hepatitis virus infection, analgesics, antibiotics, or antiemetics. After treatment, AST levels in the two groups were increased, while ALT levels were decreased (*P* < 0.05, Table 2). These results indicate that chemotherapy-assisted psychological nursing intervention combined with traditional Chinese medicine decoction can alleviate liver injury.

### 3.3. Comparison of Immunoglobulin Levels before and after Treatment in the Two Groups

Before treatment, there was no significant difference in IgG, IgA, and NK cells between the two groups (*P* > 0.05, Figure 2). After treatment, IgG and IgA in both groups were significantly decreased, and NK cells were significantly increased. The IgG and IgA of the observation group were lower than those of the control group. NK cells were higher than the control group (*P* < 0.05, Figure 2). It is suggested that traditional Chinese medicine can improve the immune function of EC patients undergoing chemotherapy.

### 3.4. Comparison of the Immune Function of the Two Groups

There was no significant difference in the levels of CD3+, CD4+, and CD8+ between the two groups before treatment. After treatment, the levels of CD3+ and CD4+ in the two groups were increased. The increase in the observation group was greater than that in the control group (*P* < 0.05, Figures 3(a) and 3(b)). Compared with before treatment, the CD8+ levels in both groups were decreased. The decrease in the observation group was significantly higher than that in the control group (*P* < 0.05, Figure 3(c)). These results also suggest that Chinese medicine can improve the immune function of EC patients undergoing chemotherapy.

### 3.5. Comparison of TCM Syndrome Scores before and after Treatment in the Two Groups

Before treatment, there was no significant difference in TCM syndrome scores between the observation group and the control group (*P* > 0.05, Table 3). After treatment, TCM syndrome scores in both groups were decreased. The observation group was lower than the control group (*P* < 0.05, Table 3). It is suggested that the combined treatment of traditional Chinese medicine can further improve the clinical symptoms. In terms of the total integral value, the improvement rate of patients in the observation group (92.34%) was significantly higher than that in the control group (85%). This may be because *Astragalus* and other traditional Chinese medicines in the prescription can significantly inhibit tumor cells and improve the effect of chemotherapy.

### 3.6. Comparison of QLQ-C30 Scores before and after Treatment in the Two Groups

After treatment, the physical, role, emotional, social, pain, and other functional scores of the two groups were improved. In the control group, there was no significant difference in the QLQ-C30 function scores between before and after treatment (*P* > 0.05, Table 4). The QLQ-C30 functional scores in the observation group were significantly different from those before treatment (*P* < 0.05, Table 4). The physical, role, emotional, and social function scores of the observation group were significantly higher than those of the control group (*P* < 0.05, Table 4). The pain function score was significantly lower than that of the control group (*P* < 0.05, Table 4).

### 3.7. Comparison of Anxiety, Depression Scores, VAS Scores, and Satisfaction between the Two Groups

Anxiety and depression scores were assessed using the SAS and SDS self-rating scales. The lower the score, the better. There was no significant difference in SDS and SAS scores between the two groups before treatment (*P* > 0.05, Table 5). After treatment, the SDS and SAS scores of the observation group were lower than those of the control group (*P* < 0.05, Table 5). After treatment, the VAS score of the observation group was 2.20 ± 0.73, which was significantly lower than that of the control group (3.76 ± 0.84). The total satisfaction of patients in the observation group (97.5%) was significantly higher than that of the control group (87.5%).

### 3.8. Comparison of Adverse Reactions between the Two Groups of Patients

The incidence of bone marrow transplant, gastrointestinal reactions, and peripheral neurotoxicity in the observation group after chemotherapy was significantly lower than those in the control group (*P* < 0.05, Tables 6 and 7). The incidence of hair loss in the observation group was slightly lower than that in the control group. The incidence of allergy and cardiovascular toxicity in the observation group was slightly higher than that in the control group (Tables 6 and 7).

## 4. Discussion

EC is a very common malignancy of the female reproductive system and is often associated with obesity, menstrual disorders, polycystic ovary syndrome, and infertility [32]. In recent years, the incidence of EC has continued to increase. The patient did not show typical clinical symptoms in the early stage of EC. When the body is unwell, it has developed to the middle and advanced stages [33]. Surgery is the first choice for the clinical treatment of EC. Drug therapy such as chemotherapy is an important part of consolidating the curative effect. If the patient is at risk, adjuvant pelvic radiation radiotherapy, systemic chemotherapy, and hormone therapy are required to control the disease [34]. However, due to the side effects of chemotherapy drugs, patients have a series of adverse reactions, which is not conducive to long-term treatment. Therefore, the treatment model of integrated Chinese and Western medicine has been gradually proposed and explored [35].

The treatment of malignant tumors with traditional Chinese medicine has been recorded as early as in the Chinese medical code of traditional Chinese medicine. However, the current curative effect detection methods and cure standards of traditional Chinese medicine cannot reflect the advantages of traditional Chinese medicine in the treatment of malignant tumors. Since the 1990s, patient clinical quality of life has been regarded by the world as a core criterion of treatment. Promoting the quality of life of patients has become the main clinical standard of TCM clinical treatment. After taking the clinical life quality of patients as the core standard for evaluating the therapeutic effect, it can better reflect the curative effect of Chinese medicine on patients. Therefore, observing the life quality of patients is used as an evaluation of the clinical therapeutic effect of traditional Chinese medicine decoction.

Conventional surgery and chemotherapy are effective treatments for EC patients. However, surgery, chemotherapy, and radiotherapy can also damage a patient's health. The operation took away the patient's blood and essence, and the radiotherapy and chemotherapy made the patient's complexion even more damaged. Therefore, EC patients experience symptoms of blood and internal organ damage after postoperative chemotherapy. Patient blood loss naturally greatly reduces the patient's quality of life. The use of traditional Chinese medicine decoction can strengthen blood of EC patients, improve the immunity of patients, and effectively prevent the recurrence and metastasis of tumor cells.

After surgery and chemotherapy, the patient's complexion began to improve, and the quality of life was improved through psychological intervention and adjuvant treatment with Chinese medicine decoction. The total effective rate and total satisfaction in the observation group were significantly higher than those in the control group. Bad mood scores were lower than the control group. The results confirmed that adjunctive therapy with Chinese herbal decoction can reduce pain and improve comfort and coordination. It can also effectively maintain white blood cell count levels, enhance resistance and tolerance, and improve patient survival. Traditional Chinese medicine decoction can help the body's immune system to perform normal postoperative self-regulation, thereby directly reducing the recurrence and metastasis rates after chemotherapy, consolidating the effect of chemotherapy, and improving prognosis (Figure 4). However, the sample size of this study is still small. In the future, our conclusions need to be further confirmed by increasing the sample size.

## 5. Conclusion

In summary, traditional Chinese medicine decoction can effectively improve the clinical therapeutic effect of EC patients undergoing chemotherapy. Chinese medicine decoction can effectively maintain immune function and tolerance and reduce toxic and side effects. In addition, Chinese medicine can relieve pain and other discomfort, improve quality of life, increase satisfaction, and prolong survival of EC patients.

## Figures and Tables

**Figure 1:** Changes in the levels of tumor markers HE4 and CA125 in the two groups. ^*∗*^*P* < 0.05, comparison before and after treatment. ^#^*P* < 0.05, comparison between the two groups after treatment.

**Figure 2:** Comparison of immunoglobulin levels before and after treatment in the two groups. ^*∗*^*P* < 0.05, comparison before and after treatment. ^#^*P* < 0.05, comparison between the two groups after treatment.

**Figure 3:** Comparison of CD3+, CD4+, and CD8+ levels between the two groups.

**Figure 4:** Chinese herbal decoction combined with psychological care can improve the clinical symptoms, alleviate side effects, and improve the life quality of EC patients with postoperative chemotherapy.

**Table 1:** Comparison of general clinical data between the two groups of patients (*n*).

Features	Observation (*n* = 40)	Control (*n* = 40)
Age (year)	43.8 ± 3.5	44.5 ± 3.9
Weight (kg)	58.3 ± 4.1	57.7 ± 4.0
Previous surgery history	9 (22.5%)	7 (17.5)
Pathological classification		
Endometrial squamous cell carcinoma	7 (12.5%)	8 (20.0%)
Endometrial cancer	33 (82.5%)	32 (80.0%)
Tumor stage		
1	6 (15.0%)	5 (12.5%)
2	17 (42.5%)	18 (45.0%)
3	14 (35.0%)	15 (37.5%)
4	3 (7.5%)	2 (5.0%)

**Table 2:** Changes in blood routine and liver function between the two groups.

Features	Control group		Observation group	
	Before	After	Before	After
Weight (kg)	58.23 ± 8.43	57.91 ± 8.17	61.46 ± 9.68	61.14 ± 10.11
WBC	5.75 ± 2.43	5.18 ± 2.75	5.56 ± 2.11	5.74 ± 2.74
RBC	11.68 ± 1.36	11.93 ± 1.61^*∗*^	12.03 ± 1.49	12.35 ± 1.51
Platelet	222.94 ± 99.87	197.45 ± 87.71	217.09 ± 92.31	227.15 ± 101.38
Creatinine	0.67 ± 0.14	0.66 ± 0.15	0.69 ± 0.21	0.67 ± 0.17
AST	27.23 ± 14.52	24.19 ± 11.01^*∗*^	27.36 ± 13.32	30.31 ± 12.85
ALT	25.68 ± 16.13	35.02 ± 20.63^*∗*^	24.12 ± 20.03	19.17 ± 10.08

^*∗*^ *P* < 0.05, compared with the control group.

**Table 3:** Comparison of TCM syndrome scores before and after treatment in 2 groups.

Group	Time	Cold pain in the abdomen	Shortness of breath	Vaginal bleeding	Sore waist and knees	Tired
Observation	Before	3.90 ± 0.52	4.18 ± 0.68	4.27 ± 0.76	3.93 ± 0.54	4.21 ± 0.41
	After	0.72 ± 0.26^*∗*^	0.71 ± 0.37^*∗*^	0.82 ± 0.47^*∗*^	0.73 ± 0.21^*∗*^	0.82 ± 0.17^*∗*^

Control	Before	3.84 ± 0.54	4.24 ± 0.68	7.31 ± 0.69	3.86 ± 0.45	4.11 ± 0.38
	After	1.30 ± 0.32	1.15 ± 0.31	1.41 ± 0.58	1.27 ± 0.34	1.37 ± 0.27

^*∗*^ *P* < 0.05, compared with the control group.

**Table 4:** Changes in quality of life in the 2 groups before and after treatment.

Group	Item	Before treatment	After treatment
Observation	Physical function	67.67 ± 5.20	73.97 ± 5.64^*∗*^
	Role function	47.61 ± 11.47	52.19 ± 10.31^*∗*^
	Emotional function	57.89 ± 12.86	63.65 ± 12.04^*∗*^
	Social function	47.72 ± 12.25	53.24 ± 11.47^*∗*^
	Pain function	24.39 ± 11.31	22.97 ± 8.42^*∗*^

Control	Physical function	67.76 ± 5.23	70.46 ± 5.36
	Role function	47.71 ± 11.52	65.64 ± 12.37
	Emotional function	57.92 ± 12.45	66.14 ± 12.73
	Social function	47.68 ± 12.03	61.83 ± 12.03
	Pain function	24.75 ± 9.29	19.15 ± 7.32

^*∗*^ *P* < 0.05, compared with the control group.

**Table 5:** Comparison of negative emotions in the two groups.

Group	Before treatment		After treatment	
	SDS score	SAS score	SDS score	SAS score
Observation	55.9 ± 3.6	53.9 ± 3.1	32.7 ± 2.3	31.2 ± 2.3
Control	56.3 ± 3.9	53.3 ± 3.3	36.3 ± 2.7	42.9 ± 3.9

**Table 6:** Adverse reactions in the observation group (*n* = 40).

Adverse reactions	0	I	II	III	IV	Incidence (%)
Bone marrow transplant	19	8	6	7	0	52.5
Gastrointestinal reactions	18	10	7	5	0	55
Peripheral neurotoxic	27	10	3	0	0	32.5
Hair loss	29	9	2	0	0	27.5
Allergy	35	4	1	0	0	12.5
Cardiotoxicity	32	5	3	0	0	20.0

**Table 7:** Adverse reactions in the control group (*n* = 40).

Adverse reactions	0	I	II	III	IV	Incidence (%)
Bone marrow transplant	10	14	8	8	0	75.0
Gastrointestinal reactions	12	14	9	5	0	70.0
Peripheral neurotoxic	20	13	5	2	0	50.0
Hair loss	21	11	7	1	0	47.5
Allergy	29	7	4	0	0	27.5
Cardiotoxicity	28	9	3	0	0	30.0

## Data Availability

The data used to support the findings of this study are available from the corresponding author upon request.
